# The use of deep learning algorithm and digital media art in all-media intelligent electronic music system

**DOI:** 10.1371/journal.pone.0240492

**Published:** 2020-10-19

**Authors:** Yingming Zheng

**Affiliations:** School of Drama and Film, Jilin University of Arts, Changchun, China; University College London, UNITED KINGDOM

## Abstract

In the development of digital media art, to explore the preliminary application of deep learning method in intelligent electronic music system, and promote the integration of deep learning method and digital media technology, thus providing a direction for the development of all media intelligent system, based on deep deterministic policy gradient (DDPG), to solve the multi-task problem in intelligent system, a multi-task learning-based DDPG algorithm (M-DDPG) is proposed. Furthermore, a DDPG algorithm based on hierarchical learning (H-DDPG) is proposed for the hierarchical analysis of images in intelligent system. Aiming at the problem of image classification in intelligent system, through the setting of simulation environment, the application effect of several algorithms in intelligent electronic music system is evaluated. The results show that: M-DDPG algorithm can more accurately complete the operation of related tasks, the reward received by the intelligent system is more than 0.35, and the test results based on eight tasks are more accurate and effective. Even in the case of task error, the algorithm still shows good training results. H-DDPG algorithm has good effect for complex task processing. The accuracy rate of task test corresponding to intelligent system in different scenarios is above 95%, which is better than other conventional algorithms in task test; the self-reinforcement network algorithm can promote the improvement of image classification effect. Several algorithms proposed show excellent performance in image processing of intelligent system, and have great application potential.

## 1. Introduction

In recent years, as computer information technology and artificial intelligence (AI) develop fast, the combination of traditional media and digital media has become increasingly close. Information not only develops from material media to digital media, but also develops from single media to multimedia and all media [1, 2]. In the development process of digital media art, electronic music is one of the typical representatives [3]. In the current context of all media, if electronic music is combined with digital media art, it will certainly play a leading role in forming new art forms. The development of digital technology is inseparable from promoting new technologies. For instance, the development of methods such as deep learning has brought opportunities for the development of digital technology, and thus promoted the intelligent development of electronic music [4–6].

For intelligent music system, scholars have carried out corresponding studies. Williams et al. (2017), through designing the emotional-driven algorithm composition and applying 16-channel feedforward artificial neural network, found that the system could create short music sequences and effectively improve the emotional range in the stimulus set composed of real world and traditional music extracts [7]. Su et al. (2017) proposed a new multimodal music recommendation system. The system integrated social information and collaborative information to predict user preferences, and it was found that the intelligent music recommendation system had superior performance [8]. Lin et al. (2019) designed and developed an intelligent motion guidance system based on music beat guidance, tested the effectiveness of the system by using quadratic polynomial regression model based on signal denoising algorithm, and found that the system had good effect in motion guidance [9]. Fakhrhosseini and Jeon (2019) proposed an emotional intelligence system based on music regulation and found that multimodal perception could be effectively applied to the overall evaluation of driver’s emotional state. Meantime, music, as a possible multimodal strategy, could reduce the impact of anger on driving performance and driver’s subjective experience [10]. Kim et al. (2020) evaluated the application of deep transfer learning method in the field of music information retrieval, and provided certain reference for the design of deep data method in music field by considering multiple target data sets [11]; Jia et al. (2019) based on downbeat tracking problem, introduced the structure of music system, feature extraction, deep neural network algorithm, data set, and evaluation strategy, providing direction for related research of music information retrieval [12]; Song et al. (2018) proposed an automatic annotation algorithm based on deep recurrent neural network, and applied it to music information retrieval. The results showed that the method had faster training speed and less memory consumption [13]; Baro et al. [14], based on convolution recurrent neural network, put forward a complete handwritten music recognition system, which is expected to realize the conversion of music score image into computer-readable format. To sum up, there are many studies on intelligent music, but the intelligent electronic music is rarely discussed. And there are many studies on the application of deep learning in the field of music information retrieval, but few on the application of deep learning to intelligent electronic music system.

Based on this, in order to expand the application of deep reinforcement learning and deep learning in intelligent electronic music system, deep deterministic policy gradient based on multi-task learning (M-DDPG) and DDPG based on hierarchical learning (H-DDPG) are introduced. Moreover, the adaptive network algorithm is applied in it, and the application effect of several algorithms in intelligent system is evaluated. This study aims to promote the integration of deep learning and digital media art, and provide a feasible direction for the development of all-media intelligent electronic music system.

## 2. Method and experiment

### 2.1 DDPG algorithm and optimization based on deep learning

In recent years, the rapid development of deep learning that has good generalization performance and feature extraction performance makes the technology widely used in many fields [15, 16]. The rise and development of reinforcement learning enables intelligent systems to complete specific tasks in specific environments through learning. It can be said that this is an effective means to promote the continuous development and optimization of intelligent systems [17]. Based on the excellent characteristics of deep learning and reinforcement learning, it is believed that the combination of deep learning and reinforcement learning can promote the performance of intelligent system. In the deep reinforcement learning algorithms, DDPG is one of the algorithm tools firstly used in continuous space regulation. This algorithm overcomes the limitations of deep Q network (DQN) algorithm in the processing of multi-action number. In addition to inputting the initial task image, it can also solve the multi-action task problem [18, 19]. Compared with DQN algorithm, there are also policy network *θ*^*π*^ and value network *θ*^*Q*^ in DDPG algorithm. In the training process of the algorithm, the corresponding minimum loss function is expressed and calculated as Eq (1).

$$L(\theta^{Q})={\left(Q(S_{t},A_{t}|\theta^{Q})-y_{t}\right)}^{2}$$ (1)

In Eq (1), *y*_*t*_ represents the supervision signal corresponding to each component sample, and *S*_*t*_ and A_*t*_ correspond to the variable, which are calculated as Eq (2).

$$y_{t}=r_{t}+\gamma Q(S_{t+1},\pi (S_{t+1}|\theta^{\pi ,t})|\theta^{Q,t}).$$ (2)

In Eq (2), *θ*^*Q*,t^ represents the target value network, *θ*^*π*,t^ indicates the target policy network, and *γ* is the parameter.

The corresponding update of *θ*^*Q*^ in the algorithm can be expressed as Eq (3).

$$\theta^{Q\prime }=\theta^{Q}-u_{Q}\cdot \nabla_{\theta^{Q}}L(\theta^{Q})$$ (3)

Furthermore, *θ*^*π*^ can complete the corresponding updating according to the gradient information obtained after the update processing, expressed as Eq (4).

$$\theta^{\pi \prime }=\theta^{\pi }-u_{\pi }\cdot \nabla_{A}Q(S_{t},\pi (S_{t}|\theta^{\pi })|\theta^{Q})\cdot \nabla_{\theta^{\pi }}\pi (S_{t}|\theta^{\pi })$$ (4)

In Eq (4), *u* is a parameter.

On this basis, the DDPG algorithm is further optimized and improved. Specifically, it is different from the single value network and single strategy network of the conventional DDPG algorithm. When improving and optimizing the DDPG algorithm, the structure corresponding to the single value network and multiple strategic networks is selected, which is proposed based on the processing of multi-task problems in intelligent system. The DDPG algorithm based on multiple policy networks is recorded as M-DDPG algorithm. To ensure the optimal update of multiple policy networks under the premise of only one value network, it needs to synchronously output the action value, Q value, corresponding to all policy networks, and the measurement standard should correspond to the task corresponding to the policy network. Additionally, due to the adoption of multiple policy networks, the parameters are increased. In order to reduce the number of parameters, mlpconv network layer is applied [20]. Compared with the conventional convolution layer, the output of the feature map corresponding to the network layer has a higher expression level. Therefore, the network layer is combined with global mean pooling, which can effectively reduce the number of parameters. Moreover, the combination of mlpconv network layer and global mean pooling can make the whole learning process of intelligent system free from interference information, and the information expressed by sensors is more intuitive. The fusion of sensor and image processing can effectively speed up the learning process, and mlpconv network layer also shows excellent performance. Fig 1 shows the overall implementation of M-DDPG algorithm. Specifically, the parameters such as the maximum number of exploration rounds, the maximum number of steps per round, the amount of batch data, memory pool, and noise intensity are input first, and then the network parameters and the target network parameters are initialized. After the number of current rounds and the number of steps are judged, the corresponding action A_t_ is output according to the decision of the policy network and the noise change, and then the action A_t_ is executed. Receive the return rt and transfer it to the next state S_t+1_; store and process the above-mentioned information such as return. Then, a batch of data is randomly selected from the stored data, and the network composition parameters and target network composition parameters are updated.

**Fig 1:** The overall implementation process of M-DDPG algorithm.

After improvement and optimization, the loss function of the value network corresponding to M-DDPG can be expressed as Eq (5).

$$L(\theta^{Q})=\sum_{n=1}^{N}{\left(Q_{n}(S_{t},{\text{A}}_{t}|\theta^{Q})-y_{n,t}\right)}^{2}$$ (5)

In Eq (5), *n* represents the number of the corresponding task and *N* corresponds to the total number of tasks. Similarly, the supervision signal changes accordingly, which can be expressed as Eq (6).

$$y_{n,t}=r_{n,t}+\gamma Q_{n}(S_{t+1},\pi (S_{t+1}|\theta^{\pi ,t})|\theta^{Q,t})$$ (6)

The gradient update of policy network can be expressed as Eq (7).

$$\nabla \theta^{\pi n}=u_{\pi n}\cdot \nabla_{A}Q_{n}(S_{t},\pi_{n}(S_{t}|\theta^{\pi n})|\theta^{Q})\cdot \nabla_{\theta^{\pi n}}\pi_{n}(S_{t}|\theta^{\pi n})$$ (7)

Finally, the update of the target network can be expressed as Eq (8).

$$\theta_{t+1}^{t}=(1-\vartheta )\theta_{t}^{t}+\vartheta \theta_{t}$$ (8)

In Eq (8), *ϑ* denotes the update factor.

Aiming at the hierarchical analysis of images in intelligent system, the M-DDPG is further extended. Specifically, the composition structure of the algorithm based on hierarchical learning includes two value networks and multiple policy networks. Compared with M-DDPG algorithm, the value network in the algorithm guides basic work and regulates complex tasks. The first layer is the base value network, and the second layer is the meta value network. The strategy network is still the learning module for each basic action. In this part, the optimized DDPG algorithm is recorded as H-DDPG. Fig 2 shows the overall implementation of H-DDPG algorithm. The H-DDPG algorithm based on AHP is actually an extension of M-DDPG algorithm. Its overall implementation process is different from M-DDPG in that the level of meta value network is higher, and other operations such as initialization and update of network parameters are consistent. In H-DDPG algorithm, the minimum cost function corresponding to the meta value network can be expressed as Eq (9).

**Fig 2:** Overall implementation process of self-reinforcement network algorithm.

$$L(\theta^{Qh})={\left(Q_{h}(S_{t},\pi_{n}(S_{t}|\theta^{\pi n})|\theta^{Qh})-y_{h,t}\right)}^{2}$$ (9)

The supervision signal can be expressed as Eq (10).

$$y_{h,t}=r_{h,t}+\gamma_{h}\underset{\pi_{n}}{\text{max}}Q_{h}(S_{t+1},\pi n(S_{t+1}|\theta^{\pi_{n}})|\theta^{Q_{h}^{t}})$$ (10)

In the H-DDPG algorithm, the final update of the target network is the same as M-DDPG algorithm.

### 2.2 Self-reinforcement network algorithm based on feature decision

To explore the image classification processing in intelligent system, self-reinforcement network algorithm is introduced, which consists of image classification network and feature decision-making intelligent system. Under the collaborative processing of these two parts, image classification process can be realized [21]. Fig 2 shows the overall implementation process of the algorithm.

The image classification network is the core of the algorithm, which is mainly composed of two modules: feature pre-extraction and feature extraction. The former mainly includes two convolution layers, which can reduce the dimension of the corresponding image and the amount of calculation; the latter mainly consists of DenseBlock, which can realize the extraction of high-dimensional features of corresponding images and provides reference for image classification. Feature decision-making intelligent system is an important component of self-reinforcement, which can evaluate the image states. The module contains several important elements, among which action and return function are the cores. In the feature space formed by the classification dataset, the intelligent system is expected to achieve better image classification and optimize the related features. In the self-reinforcement network algorithm, the intelligent system can make the image classification network focus on the input image through transforming the corresponding image, thus getting more accurate classification results. Additionally, mlpconv network layer [22] is still used to achieve feature output. The feature decision-making intelligent system takes the relevant reward information received as the basis, and then conducts strategy learning. In this algorithm, the confidence level which can be correctly identified is used as the evaluation index. If the confidence increases, the system will receive a positive return; if the confidence decreases, the system will receive a negative return. Specifically, it can be expressed as Eq (11).

$$r_{t}=\{\begin{array}{cc} r_{A}, & P_{t}(C_{t})>P_{t-1}(C_{t})\\ -r_{A}, & P_{t}(C_{t})\leq P_{t-1}(C_{t}) \end{array}$$ (11)

In Eq (11), *P*_*t*_ represents a certain type of confidence corresponding to the current action time, and *C*_*t*_ suggests the real category, and *r*_*A*_ corresponds to the specific return value. The corresponding relationship between return value and strategy and ordinary action can be expressed as Eq (12).

$$r_{t}=\{\begin{array}{cc} r_{e}, & \underset{C}{\text{max}}P_{t}(C)=C_{t}\\ -r_{e}, & \underset{C}{\text{max}}P_{t}(C)\neq C_{t} \end{array}$$ (12)

In Eq (12), *r*_*e*_ refers to the specific return value under the current situation. In other words, in the final action, if there is no fault in the classification of the image, the system will receive a positive return; otherwise, it will be a negative return. In the intelligent system of the algorithm, the optimization of the corresponding action Q value can be expressed as Eq (13).

$$L(\theta^{Q})={\left(Q(S_{t},A_{t}|\theta^{Q})-y_{t}\right)}^{2}$$ (13)

The supervision signal is expressed and calculated as Eq (14).

$$y_{t}=r_{t}+\gamma \underset{A_{t+1}}{\text{max}}Q(S_{t+1},{\text{A}}_{t+1}|\theta^{Q^{t}})$$ (14)

### 2.3 Construction of all-media intelligent electronic music system based on digital media art

As the digital media develops and popularizes, digital art is gradually changing to multimedia, mixed media, and all media. In this process, the application of AI tools in the field of digital art has also been developed. In the construction of all-media intelligent electronic music system, the data operation of image and action information is one of the key links, and the deep learning method shows excellent performance in the application of image processing. Based on this, the M-DDPG algorithm, H-DDPG algorithm, and self-reinforcement network algorithm are applied to the operation and processing of image and action information of all-media intelligent electronic music system. For constructing the intelligent system, the computer automatic composition system is taken as an example. The system integrates the deep reinforcement learning algorithm and the deep learning algorithm composition into it. Combined with the interactive design, the two digital art creation modes are applied. When the computer is used to complete the automatic creation, the related variables and parameters are interfered by the interactive method. In this context, people’s subjective initiative and the organic feedback of the object can ultimately realize the creation of electronic music. In the construction of the all-media intelligent electronic music system, deep intelligent learning algorithm, image, action, and interactive information are combined. Moreover, the image and action information data processing subsystem of the intelligent system is emphasized.

Fig 3 suggests the overall functional structure of the all-media intelligent electronic music system and the working mode of the all-media intelligent electronic music creation subsystem based on image and action information processing. In this system, sensor-based behavior sensing and computer-based music motivation generation are the key links, which correspond to the music generation conditions in the subsystem. Based on this, the output of sound signal and data information in the system can be completed.

**Fig 3:** Function realization of all-media intelligent electronic music system.

### 2.4 Experimental setting

To verify the effect of deep intelligent learning algorithm in the all-media intelligent electronic music system, a simulation environment is established, which is formed by the barrier-free space surrounded by all directions. The establishment and description of such a simulation environment is actually a kind of simulation operation of the musical note beating in the electronic music system. The overall presentation of music performance is in an open space, so the simulation space constructed is barrier-free space. In this space environment, suppose that there is a robot car running freely, and each action in the process of computer automatic composition is compared to the movement of a machine car. Meantime, to master the source of image information of deep learning algorithm, the real-time image information is obtained by installing a camera in front of the robot car; the speed of the machine car in different action states is mastered by the sensor. In the all-media intelligent electronic music system, depending on the input image information and the real-time information provided by the sensor, the specific action state can be selected and a specific task can be completed.

In the performance verification of deep learning algorithms M-DDPG and H-DDPG, the specific network structure parameters are set as follows: in the M-DDPG algorithm, the mlpconv network in the first layer outputs 32 characteristic graphs, the size of the outermost convolution kernel is 8*8, and the step size is 4. Then, the corresponding feature map output of the back-convolution layer is 64, the size of the convolution kernel is 4*4, and the step size is 2. In the last mlpconv network layer of convolution layer, the corresponding feature map output is 64, the size of convolution kernel is 3*3, and the step size is 1. The value network is composed of two layers of fully connected layers, and the number of nodes corresponding to the two full connection layers is 400 and 300 respectively. The policy network is also composed of two layers of fully connected layers, and the corresponding number of nodes is 300 and 200, respectively. The output of the number of nodes corresponding to the value network corresponds to the Q value of the task, while the policy network outputs the action decision of the corresponding task. The network training is completed in TensorFlow platform.

In the verification and training of H-DDPG algorithm performance, in the same simulation environment as above, three different scenarios are selected for experiment. In each composition scenario, there is a complex task to be completed by intelligent system. Specifically, the three scenes are adjacent to the object, adjoining the specified target, and leaving the location of the specified target. For the setting of relevant parameters, the first layer of convolution layer has 32 corresponding feature maps, the size of convolution kernel is 8*8, and the corresponding step size is 4; the corresponding parameters of the second layer are 64, 4*4 and 2, and those of the third layer are set as 64, 3*3, and 1, respectively. For the fully connected layer, the number of nodes corresponding to the two layers of the meta value network is 512 and 256, and that of the base value network is both 300, and that in the strategy layer are 200 and 150, respectively.

## 3. Results

### 3.1 Multi-task learning performance of M-DDPG algorithm

The music note beat in the intelligent electronic music is simulated as a robot car. In the learning state of six tasks, the robot car control based on the all-media intelligent electronic music system is implemented, and Fig 4 shows the results.

**Fig 4:** Performance test results of M-DDPG algorithm under 6 tasks (A represents backward action state, F represents forward, F-R represents forward-right turn, F-L represents forward-left turn, A-R represents backward-right turn, A-L represents backward-left turn).

The data changes in Fig 4 suggests that under the learning of six tasks, M-DDPG algorithm can operate the corresponding tasks more accurately, and the rewards received by the intelligent system are all above 0.35. It indicates that the returns that the intelligent system receives are all positive, which also reflects the accuracy of task processing. The learning effect of M-DDPG algorithm in multi-task setting is excellent.

Under the premise of eight tasks, the performance of M-DDPG algorithm and DDPG algorithm is tested and compared, as shown in Fig 5(a) and 5(b).

**Fig 5:** Performance test results of M-DDPG algorithm under 8 tasks (A-D represents fast straight forward, fast-forward-right turn, fast-forward-left turn, and fast straight backward; E-H respectively represents slow straight forward, slow-forward-right turn, slow-forward-left turn, and slow straight backward).

The data changes in Fig 5 indicates that the performance of M-DDPG algorithm in each task is equivalent to that of single DDPG algorithm in intelligent system. Meanwhile, comparing the performance test results based on eight tasks with that based on six tasks, it can be found that whether the number of tasks is large or small and whether the difficulty of tasks increases, it does not greatly affect the final results. Whereas, the test results based on eight tasks are obviously more accurate, which further reflects the effectiveness of M-DDPG algorithm in all-media intelligent electronic music system.

Based on the former test, a wrong task is added by setting the return function corresponding to the task to 0 or 1, thereby further testing the performance of M-DDPG algorithm. Fig 6 shows the corresponding test results.

**Fig 6:** Performance test results of M-DDPG algorithm when adding an error task (Fs represents the error strategy).

Fig 6 illustrates that even in the case of learning failure caused by task errors, M-DDPG algorithm can also train the corresponding tasks well.

### 3.2 Performance test of H-DDPG algorithm

Fig 7 shows the test results of base value network performance of H-DDPG algorithm in three different scenarios.

**Fig 7:** Performance test results of the base value network in H-DDPG algorithm under three scenarios (L- represents the action state to the left, R- to the right, and 1, 2, and 3 denote scenario 1, 2, and 3, respectively).

The data information in Fig 7 reveals that in three different scenarios, the strategy network corresponding to four different actions can show excellent performance after about 1500 exploration rounds, and the performance can be maintained relatively stable. Compared with M-DDPG, the performance of H-DDPG is slightly worse, but this is also related to the actual environment of H-DDPG.

Fig 8 shows the performance test results of the meta value network of H-DDPG algorithm in three different scenarios.

**Fig 8:** Performance test results of meta value network in H-DDPG algorithm under three scenarios.

Fig 8 indicates that the intelligent system gradually finds the strategy and method of task solving after about 2000 exploration rounds. Corresponding to scenario 1 and scenario 2, after the whole training process is relatively stable, the accuracy rate of task test of intelligent system is above 90%, that of scenario 3 is about 80%. However, scenario 3 shows completely different changes from scenario 1 and scenario 2. When the number of exploration rounds reaches 6000, the overall training process achieves a relatively stable change, the corresponding task success rate is also low, and the overall task test accuracy reaches 87.6%.

Fig 9 shows the comparison of optimal test results between H-DDPG algorithm and other algorithms.

**Fig 9:** Comparison of optimal test results between H-DDPG algorithm and other algorithms.

Fig 9 suggests that, corresponding to three different scenarios, H-DDPG algorithm shows the best performance, with an average success rate of 95%. In contrast, the average success rate of DQN algorithm is 66.67%, and that of DDPG algorithm is only 16.67%.

### 3.3 Performance of self-reinforcement network algorithm based on image classification and enhancement

In the application of self-reinforcement network algorithm in intelligent system, the number of corresponding output actions and the corresponding distribution change of correct number under different action execution time are shown in Fig 10.

**Fig 10:** The output quantity of actions and their corresponding distribution changes of correct number under different action execution times.

Fig 10 reveals that, corresponding to the execution time of each different action, the accuracy corresponding to the output image in the final intelligent system is maintained high, and the more the corresponding classification number is, the higher the classification accuracy rate is. It means that the intelligent system can effectively classify the current image according to the feature map.

## 4. Discussion

The above analysis indicates that the learning effect of M-DDPG algorithm in multi-task setting is excellent, and the number of tasks or the difficulty level of tasks will not affect its final robust performance. Each strategy network in the algorithm can learn the corresponding task strategy in the early stage of training, and can maintain the performance. In the first 1000 exploration rounds, the corresponding return has a great change, which is mainly because the car’s motion is not stable enough in the initial stage but fluctuates. The major reason is that the shared parameters between different networks and the shared memory pool between different tasks enable the intelligent system to receive more positive return data, and meantime, it increases the warning of wrong actions. The strategy gradient calculation corresponding to M-DDPG algorithm reduces the interference between the gradients with different policy networks, thus enhancing the robustness of the algorithm, even showing excellent performance in the wrong task. In a word, M-DDPG algorithm has excellent robustness in multi-task learning. It can not only effectively reduce the number of parameters, but also has good scalability. Therefore, it has great application potential in the multi-task intelligent electronic music system, especially for image and motion processing.

In the continuous "action" space such as electronic music composition, H-DDPG algorithm can achieve efficient learning for complex tasks. Hierarchical learning based on deep learning has excellent performance in learning complex tasks. The low success rate of corresponding tasks in scenario 3 may be caused by the friction between the robot car and the side of the door in the simulation environment. The overall success rate of the algorithm in task processing is high. Compared with other conventional algorithms based on discrete action space, H-DDPG algorithm shows significant advantages, which further verifies the effectiveness of H-DDPG algorithm in all-media intelligent electronic music system. The application of feature decision-making intelligent system in self-reinforcement network algorithm can promote the accuracy of image recognition network. The specific settings in the algorithm also provide a favourable premise for image classification and enhancement, but it may be affected by strategy or action transformation, so the algorithm is not very ideal in improving the confidence of image category. But even so, the application of the self-reinforcement network algorithm still has a very significant effect on improving the image processing ability of all-media intelligent electronic music system.

## 5. Conclusion

The performance of M-DDPG algorithm based on image multi task learning, H-DDPG algorithm based on image hierarchical analysis, and adaptive reinforcement network algorithm based on image classification is analysed. It is found that M-DDPG has good robustness and H-DDPG algorithm has applicability in multi-task complex environment. Adaptive reinforcement network algorithm can effectively promote image classification and enhancement, which provides a certain experimental reference for the application of degree learning in intelligent electronic music system. However, the application of deep learning algorithm in the all-media intelligent electronic music system under digital media art is still in the initial stage of exploration, so there are still some shortcomings. This research only analyzes the image and motion processing module subsystem of the intelligent system, the proposed image processing algorithms still need to be optimized, and the future research will focus on other functional modules in the intelligent system.

## Supporting information

S1 File (ZIP)
